The article "MeCP2 drives hepatocellular carcinoma progression via enforcing HOXD3 promoter methylation and expression through the HB‐EGF/EGFR pathway" was retracted in 2024. Reasons: duplicated images; unreliable data; unreliable results or conclusions.

# MeCP2 drives hepatocellular carcinoma progression via enforcing *HOXD3* promoter methylation and expression through the HB‐EGF/EGFR pathway

**DOI:** 10.1002/1878-0261.13019

**Published:** 2021-06-10

**Authors:** Lumin Wang, Yi Gao, Dongdong Tong, Xiaofei Wang, Chen Guo, Bo Guo, Yang Yang, Lingyu Zhao, Jing Zhang, Juan Yang, Yannan Qin, Liying Liu, Chen Huang

**Affiliations:** ^1^ Department of Digestive Diseases in Precision Medicine Institute the Second Affiliated Hospital of Xi'an Jiaotong University China; ^2^ Department of cell Biology and Genetics School of Basic Medical Sciences Xi'an Jiaotong University Health Science Center China; ^3^ Yan'an Key Laboratory of Chronic Disease Prevention and Research China; ^4^ Key Laboratory of Environment and Genes Related to Diseases Xi'an Jiaotong University Health Science Center China; ^5^ Institute of Genetics and Developmental Biology Translational Medicine Institute School of Basic Medical Sciences Xi'an Jiaotong University Health Science Center China; ^6^ Cardiovascular Research Center Xi'an Jiaotong University Health Science Center China

**Keywords:** HB‐EGF, HCC, HOXD3, MeCP2, methylation, progression

## Abstract

Homeobox D3 (HOXD3), a member of the homeobox family, was described to regulate tumorigenesis, invasion, metastasis, and angiogenesis in various tumor types. However, the molecular mechanisms regulating HOXD3 during hepatocellular carcinoma (HCC) migration, invasion, and angiogenesis remain elusive. In this study, we demonstrated that HOXD3 expression is enhanced by the binding of methyl‐CpG‐binding protein 2 (MeCP2), a methyl‐CpG binding protein, together with CREB1to the hypermethylated promoter of *HOXD3*. Inhibition of HOXD3 eliminated the tumorigenic effects of MeCP2 on HCC cells. Furthermore, HOXD3 directly targeted the promoter region of heparin‐binding epidermal growth factor (HB‐EGF) *via* the EGFR‐ERK1/2 cell signaling pathway and promoted invasion, metastasis, and angiogenesis of HCC *in* *vitro* and *in vivo*. Additionally, elevated expression of MeCP2, CREB1, and HB‐EGF in HCC correlated with a poor survival rate. Our findings reveal the function of the MeCP2/HOXD3/HB‐EGF regulatory axis in HCC, rendering it an attractive candidate for the development of targeted therapeutics and as a potential biomarker in patients with HCC.

## Graphical abstract

Hepatocellular carcinoma (HCC) is considered the fifth most common cancer and a frequent cause of cancer‐related death. In our study, we observed that methyl‐CpG‐binding protein 2 (MeCP2) drives HCC progression by recruiting CREB1 and enforcing *HOXD3* expression. Hypermethylation of the homeobox D3 (HOXD3) promoter *via* the heparin‐binding epidermal growth factor (HB‐EGF) signaling pathway induced invasion, migration, and angiogenesis of HCC. Our findings reveal the function of the MeCP2/HOXD3/HB‐EGF regulatory axis in HCC, rendering it an attractive candidate for the development of targeted therapeutics and as a potential biomarker in patients with HCC.

The article "MeCP2 drives hepatocellular carcinoma progression via enforcing HOXD3 promoter methylation and expression through the HB‐EGF/EGFR pathway" was retracted in 2024. Reasons: duplicated images; unreliable data; unreliable results or conclusions.

**Abbreviations**
5‐Aza: 5‐azacytidine
DSS: disease‐specific survival
EGF: epidermal growth factor
HB‐EGF: heparin‐binding epidermal growth factor
HCC: hepatocellular carcinoma
HOXD3: homeobox D3
MBD: methyl‐CpG‐binding domain
MeCP2: methyl‐CpG‐binding protein 2
MM: multiple myeloma
MVD: microvessel density
OS: overall survival
PFI: progression‐free interval event
TRD: transcriptional repression domain

## 1 Introduction

Globally, hepatocellular carcinoma (HCC) is one of the most prevalent types of tumors, representing the fifth most common human malignancy and the third highest cause of cancer‐related mortality [1]. Although the HCC death rate has decreased in the past few decades because of prevention, accuracy in diagnosis, and treatment, the overall prognosis of HCC remains low due to the high rates of tumor recurrence and the propensity for metastasis. Furthermore, the molecular mechanisms underlying angiogenesis in HCC remain largely unclear. Homeobox D3 (HOXD3), a member of the homeobox family, participates in various biological processes such as tumorigenesis, invasion, metastasis, and angiogenesis. In colorectal cancer [2], downregulation of HOXD3 expression remarkably suppressed proliferation and induced apoptosis in RKO cells. In our previous study, vitamin D3 regulated miR‐99‐3p *via* the HOXD3 signaling pathway to contribute to the antiproliferative effects of gastric cancer [3]. In a recent study on HCC, Li *et␣al*. [4] found that matrine inhibited cell progression, migration, and invasion and promoted autophagy by regulating the circ_0027345/miR‐345‐5p/HOXD3 axis. Thus, HOXD3 is key for the overall understanding of HCC progression. However, the exact effect of HOXD3 on the invasion, metastasis, and angiogenesis of HCC remains elusive.

Heparin‐binding epidermal growth factor (HB‐EGF) is a member of the epidermal growth factor (EGF) family involved in the progression of many solid tumors including malignant gliomas [5], lung cancer [6], and multiple myeloma (MM) [7]. HB‐EGF can pass through EGFR and Axl to initiate glioblastoma in mice. Additionally, HB‐EGF is highly expressed in MM patients and is a potent activator of angiogenesis in MM. In HCC, TMPRSS4 can regulate the expression of HB‐EGF to induce HCC progression [8]. The effect of HB‐EGF on HCC migration, invasion, angiogenesis, and the potential molecular regulatory mechanisms of HB‐EGF need to be investigated further, especially the relationship between HOXD3 and HB‐EGF in HCC.

The article "MeCP2 drives hepatocellular carcinoma progression via enforcing HOXD3 promoter methylation and expression through the HB‐EGF/EGFR pathway" was retracted in 2024. Reasons: duplicated images; unreliable data; unreliable results or conclusions.

Methyl‐CpG‐binding protein 2 (MeCP2) is a methyl‐CpG‐binding protein. Previous studies have identified that MeCP2, as a transcription suppressor, affects the tumor regulatory mechanism by recruiting histone deacetylases and methylases to methylated DNA. MeCP2 can bind to the methylated CpG island of genes to inhibit the expression of genes and affect the progression of cancers such as pancreatic cancer [9] and gastric cancer [10]. Recent studies have shown that MeCP2 acts as a transcription activator in gene regulation, and MeCP2 collaborates with CREB1 to induce local histone H3 acetylation, thereby counteracting inflammation‐induced epigenetic silencing of foxp3 [11]. Meanwhile, recruitment of CREB1‐MeCP2 promotes the developmental neuronal glut3 gene transcription and expression *via* banding the glut3‐CpGs [12]. In HCC, MeCP2 promotes cell proliferation by activating ERK1/2 [13]. However, compared with the MeCP2 inhibition of gene transcription, a study on the function of MeCP2 as a transcription activator in gene expression regulation is needed to confirm this in HCC.

In this study, our data revealed that MeCP2 recruits CREB1 bound to the CpGs of the HOXD3 promoter region. From the gain‐ and loss‐of‐function of MeCP2 and HOXD3, MeCP2 promoted the expression of HOXD3 *via* the HB‐EGF cell signaling pathway to induce migration, invasion, and angiogenesis in HCC. This is the first study to demonstrate the correlation between MeCP2 and HOXD3 as well as between HOXD3 and HB‐EGF. This finding indicates that the MeCP2‐HOXD3‐HB‐EGF interaction plays an indispensable role in HCC treatment.

## 2 Materials and methods

### 2.1 Human samples and HCC cell lines

Thirty‐six pairs of human HCC samples and adjacent nontumor tissues were obtained from the First Affiliated Hospital of Xi'an Jiaotong University. Informed consent was obtained from all patients, and the study was approved by the Institute Research Ethics Committee of The Cancer Center of Xi'an Jiaotong University and study methodologies conformed to the standards set by the Declaration of Helsinki. The human liver cancer lines MHCC‐97H, Huh7, and normal liver cell lines HL‐7702 were obtained from the company (Shanghai Zhong Qiao Xin Zhou Biotechnology Co., Ltd., Shanghai, China) and were cultured as previously described [14]. All cell lines were transfected with Lipofectamine 2000 (Invitrogen, Carlsbad, CA, USA) or RNAiMax transfection reagent (Invitrogen) according to the manufacturer's instructions.

### 2.2 Plasmids and siRNA

The plasmid of MeCP2, HOXD3, shMeCP2‐1, shMeCP2‐2, shHOXD3‐1, and shHOXD3‐2 Lentivirus vector was obtained from the company (GeneChem).

The article "MeCP2 drives hepatocellular carcinoma progression via enforcing HOXD3 promoter methylation and expression through the HB‐EGF/EGFR pathway" was retracted in 2024. Reasons: duplicated images; unreliable data; unreliable results or conclusions.

### 2.3 Total RNA extraction and quantitative RT‐PCR

Total RNA was isolated from the tissues and cell lines using TRIzol reagent (Invitrogen). RNA was extracted from the Huh7 cells transfected with HOXD3 and negative control and analyzed by KangChen Bio‐tech company, Shanghai, China. cDNA was synthesized by reverse transcription according to the manufacturer's instructions (Takara Biotechnology, , Takara, Dalian, China). Quantitative RT‐PCR was performed using the SYBR Green PCR kit (Takara Biotechnology). qRT‐PCR was performed according to the methods described previously, and gene expression was normalized by GAPDH. All primers used in the present research are shown in Table S1. The relative fold change in RNA expression was calculated using the 2^−ΔΔCt^ method.

### 2.4 Bisulfite sequencing PCR

The methylated level of CpG was assessed by the BSP analysis using a Bisulfite Conversion Kit (Active Motif, Carlsbad, CA, USA) according to the manufacturer's instructions. Briefly, the genomic DNA from the cells was carried out using a genomic DNA extraction Kit (Omega, Norcross, GA, USA). Bisulfite modification of 2 µg of genomic DNA was performed with a bisulfite reagent. The primers for the BSP were designed with the Methy1 Primer express program. The QUMA Analyzer online tool was used to calculate the methylation percentage.

### 2.5 Scratch wound assay

Transfected HCCs were plated to 50% confluence on six‐well plates. A pipette tip was used to form a scratch wound. The detached cells were washed with PBS and cultured in the 1% FBS fresh medium. The image was measured 0, 48 h after wounding using a Leica microscope.

### 2.6 HCCs invasion assay

Cell invasive capability was assessed by transwell assay. Briefly, 2.0 × 10^4^ cells in serum‐free DMEM were seeded into the upper chamber which was coated with Matrigel (Becton Dickinson Biosciences, Bedford, MA, USA), and the bottom chambers contained DMEM with 10% FBS. After 48‐h incubation, the remaining cells in the upper chamber were removed. Cells had passed through gel and attached to the lower surface of the membrane were stained with 1% crystal violet and photographed. Each experiment was performed in triplicate.

### 2.7 Capillary tube formation assay

*In vitro* angiogenesis was performed as previously described [15]. Briefly, transfected HUVECs (4 × 10^4^ cells per well) were plated onto 96‐well plates pre‐coated with 50 μL of Matrigel (Becton Dickinson Biosciences) and cultured in conditioned media for 8 h to assess the formation of capillary‐like structures. Capillary‐like structures were photographed, and the number of formed tube was analyzed.

The article "MeCP2 drives hepatocellular carcinoma progression via enforcing HOXD3 promoter methylation and expression through the HB‐EGF/EGFR pathway" was retracted in 2024. Reasons: duplicated images; unreliable data; unreliable results or conclusions.

### 2.8 Spheroid sprouting assay

HUVECs were transfected with MeCP2‐Ctrl, MeCP2, shMeCP2‐Ctrl, shMeCP2, HOXD3‐Ctrl, HOXD3, shHOXD3‐Ctrl, and shHOXD3. After 24‐h incubation, HUVECs were harvested. 1 × 10^5^ HUVECs were seeded to a 96‐well plate in 150 µL of ECM medium. Cells formed spheroids overnight at 37 °C. Afterward, spheroids were embedded in an equivalent solution of collagen type I from rat tail (Becton Dickinson) and incubated at 37 °C for 1 h followed by the addition of growth medium. After 72 h, the spheroids formed sprouts, which were imaged using a Leica microscope at 4 and 10× magnification.

### 2.9 Western blotting assay

Western blotting was used as previously described [16]. Protein was isolated from patient tissues and HCCs with RIPA lysis buffer with protease inhibitor (Invitrogen). Protein concentration was determined with a bicinchoninic acid protein assay kit (Beyotime). Equal amounts of protein were separated by electrophoresis in a 12.5% SDS/PAGE and transferred to a nitrocellulose membrane, and immunoblotted with specific antibodies. The protein bands were detected and analyzed by chemiluminescence and densitometric system.

### 2.10 Chromatin immunoprecipitation assay

Chromatin immunoprecipitation assay (ChIP) was performed according to the methods described previously [17]. Briefly, Huh7 cells were fixed with 1% formaldehyde for 10 min and then quenched by using glycine (0.125 mol·L^−1^) for 30 min. Nuclei lysates were sonicated using a cell cracker to generate ˜ 200 bp DNA fragments and then incubated with 10 μg CHIP grade antibodies against MeCP2, HOXD3, GFP, and IgG, respectively (Abcam, Cambridge, MA, USA), at 4 °C overnight. DNA was analyzed by qPCR. The primer sequences used are listed in Table S1.

### 2.11 Luciferase activity assays

Luciferase activity assay was performed as described in detail [18]. Briefly, Huh7 and HMCC‐97H cells were plated on 96‐well plates. Twenty‐four hours later, dual‐luciferase vector containing the WT or Mut‐specific promoter region was cotransfected with the indicated plasmids, respectively. The dual‐luciferase reporter assay (Promega, Madison, WI, USA) was performed to measure the luciferase activity according to the manufacturer's manual.

### 2.12 Immunohistochemistry

Immunohistochemistry was performed to examine MeCP2 and HB‐EGF expression in human liver cancer and nontumor tissues at protein level. Immunohistochemistry was conducted as our previous work [19].

### 2.13 Immunofluorescence microscopy

Immunofluorescence microscopy was applied to examine the location of proteins in HCCs. Immunofluorescence microscopy was used as previously described in detail [20]. Briefly, after 48 h transfected, the HCCs were fixed with 4% formaldehyde and permeabilized with 0.1% Triton X‐100. Nonspecific binding sites were blocked by incubation in 10% of normal goat serum. The cocultures were stained for Rabbit anti‐MeCP2 (Cell Signaling Technology; diluted 1/500) and mouse anti‐CREB1 antibody (Cell Signaling Technology, Boston, MA, USA; diluted 1/500), and the images were captured by a Nikon Eclipse TS100 microscope (Nikon, Tokyo, Japan).

The article "MeCP2 drives hepatocellular carcinoma progression via enforcing HOXD3 promoter methylation and expression through the HB‐EGF/EGFR pathway" was retracted in 2024. Reasons: duplicated images; unreliable data; unreliable results or conclusions.

### 2.14 Immunoprecipitation

Immunoprecipitation assay was performed as previously described [10]. Briefly, total proteins were extracted from MHCC‐97H and Huh7 cells by RIPA buffer and incubated with 3–4 μg MeCP2 and CREB1 antibodies at 4 °C overnight. Then, protein G agarose beads were added to lysates containing proteins and antibodies for 3 h. The beads were washed five times with PBS, and the samples were examined by western blotting assay.

### 2.15 Tumorigenicity assay *in vivo*

Male BALB/c nude mice (BALB/c‐Foxn1^nu^/Arc) were purchased from the animal center of Xi'an Jiaotong University. All mice were housed and treated in accordance with widely accepted standards, and the protocols were approved by the guidelines of the Animal Care and Use Committee of Xi'an Jiaotong University (animal experimental license number: 2018‐321). Construction of tumor migration mouse model was performed as previously described [18]. In brief, shMeCP2‐Ctrl‐ and shMeCP2‐transfected Huh7 cells were injected into nude mice through the tail vein (6‐week‐old). At the end of the experiment, the mice were executed, and the lungs of mice were isolated. The fixed lung was subjected to HE staining.

### 2.16 Statistical analysis

All experiments were repeated at least three times. Student's *t*‐test was performed to analyze the two groups. The ANOVA followed by Tukey's was used to compare the multiple groups. All of the data were analyzed using spss 17.0 statistical software (SPSS Inc., Chicago, IL, USA). *P* < 0.05 was considered statistically significant.

## 3 Results

### 3.1 MeCP2 more highly expressed in HCC tissues and associated with patients' overall survival

TCGA and GTEX databases were used to confirm the clinical value of MeCP2 expression in HCC tissues. MeCP2 was expressed at higher levels in HCC tissues than in normal tissues at the mRNA level (Fig. 1A). Meanwhile, the expression of MeCP2 was related to the pathological stage of HCC patient specimens (*P* = 0.008; Fig. 1B). Further analysis showed that MeCP2 expression increased gradually in the T1, T2, T3, and T4 groups (*P* = 0.045; Fig. 1C), and higher expression of MeCP2 contributed to a lower survival rate (Fig. 1D and Fig. S1A,B). MeCP2 expression was associated with overall survival (OS, *P* = 0.0056), progression‐free interval event (PFI, *P* = 0.037), and disease‐specific survival event (DSS, *P* = 0.028) of HCC. Consistent with the results from TCGA and GTEX databases, higher expression of MeCP2 was identified in HCC tissues than in normal tissues in our 36 collected paired patient samples. MeCP2 was significantly upregulated in 83% (30/36) of the HCC samples (Fig. 1E). High expression was associated with the pTNM stage of tumor samples (*P* = 0.013) (Table 1). The expression of MeCP2 at the protein level was also examined by IHC in human liver cancer tissues. Upregulation of MeCP2 was observed in HCC tissues versus normal tissues. CD34 is a marker of angiogenesis, and its expression was tested using IHC. Compared with the microvessel density (MVD) in MeCP2 normal tissue samples, we found that MVD was dramatically increased in MeCP2 overexpression patients (Fig. 1F). In addition, MeCP2 expression was also increased in the four pairs of HCC tissues (Fig. 1G). To further clarify the effect of MeCP2 in HCC, MHCC‐97H and Huh7 cell lines were analyzed. Compared with HL‐7702 cells, the expression of MeCP2 was increased in MHCC‐97H and Huh7 cells (Fig. 1H). Based on the above analysis results, MeCP2 is considered to be a tumor activator in HCCs.

The article "MeCP2 drives hepatocellular carcinoma progression via enforcing HOXD3 promoter methylation and expression through the HB‐EGF/EGFR pathway" was retracted in 2024. Reasons: duplicated images; unreliable data; unreliable results or conclusions.

**Fig. 1:** MeCP2 is more highly expressed in HCC and induces low survival rate. (A) TCGA and GTEX showed that MeCP2 higher expression in liver cancer tissues (*n* = 371) than in normal tissues (*n* = 160). Student's *t*‐test. The error bar was SD. (B) Correlation between MeCP2 expression and pathologic stage (Stage I *n* = 170, Stage II *n* = 87, Stage III *n* = 85, Stage IV *n* = 5) in HCC patients. *P* values are estimated by one‐way ANOVA. The error bar was SD. (C) The relationship between MeCP2 expression and T (T1 *n* = 180, T2 *n* = 95, T3 *n* = 80, T4 *n* = 13) stage in HCC patients. The error bar was SD. (D) MeCP2 expression was correlated with liver cancer OS. Kaplan–Meier plots and log‐rank tests were used for statistical analysis. (E) MeCP2 expression at the RNA level in 36 paired clinical samples. Student's *t*‐test. The error bar was SD. (F, G) Western blotting and IHC were performed to compare the expression of MeCP2 and CD34 in normal tissues and HCC tissues at the protein level. Scale bar: 50 μm. (H) MeCP2 expression in HL‐7702, MHCC‐97H, and Huh7 cells. Student's *t*‐test. The error bar was SEM. (*n* = 3 per group. *P < 0.05, **P < 0.001).

**Table 1:** Patient characteristics and clinicopathologic correlation of MeCP2, HOXD3 and HB‐EGF expression.

Characteristics	Number of cases	MeCP2 expression		*P*‐value	HOXD3 expression		*P*‐value	HB‐EGF expression		*P*‐value
		High	Low		High	Low		High	Low	
Age (years)										
≥ 60	16	14	2	0.672	15	1	0.104	15	1	0.053
< 60	20	16	4		14	6		13	7	
Gender										
Male	24	21	3	0.378	21	3	0.190	18	6	0.691
Female	12	9	3		8	4		10	2	
pTNM Stage										
I	11	10	1	0.013	9	2	0.021	9	2	0.947
II	10	5	5		5	5		7	3	
III	9	9	0		9	0		7	2	
IV	6	6	0		6	0		5	1	
Histology										
Well	21	19	2	0.23	20	1	0.002	18	3	0.009
Moderate	8	4	4		3	5		3	5	
Poor	7	7	0		6	1		7	0	

The article "MeCP2 drives hepatocellular carcinoma progression via enforcing HOXD3 promoter methylation and expression through the HB‐EGF/EGFR pathway" was retracted in 2024. Reasons: duplicated images; unreliable data; unreliable results or conclusions.

### 3.2 MeCP2 induces metastasis, invasion, and angiogenesis of HCCs *in vitro* and vivo

The gain‐ and loss‐of‐function of MeCP2 assays were used to explore the role of MeCP2 in HCC. MeCP2 expression was significantly upregulated in MeCP2‐transfected HCCs compared with MeCP2‐Ctrl‐transfected HCCs (Fig. S2A,B). A wound‐healing assay was used to evaluate the crucial role of MeCP2 in the migratory ability of HCCs. Transfection with MeCP2 induced a faster rate of HCC wound closure than the negative control, suggesting that MeCP2 increased the migration of MHCC‐97H and Huh7 cells (Fig. 2A and Fig. S2C). Similarly, the cell invasive ability of Huh7 and HMCC‐97H cells transfected with MeCP2 was increased compared with the blank control (Fig. 2B and Fig. S2D). Tube formation assays were used to identify the function of MeCP2 in the angiogenesis of HUVECs. The results showed that the average number of tubular structures shaped by HUVECs transfected with MeCP2 significantly increased (Fig. 2C). In addition, we generated spheroids consisting of MeCP2‐ or negative control‐transfected HUVECs and assessed their cellular sprouting capacity. Consistent with the results of the wound healing and transwell assays, MeCP2 increased the length of newly developed sprouts (Fig. 2D). To further confirm that MeCP2 plays the role of tumor activator in invasion, metastasis, and angiogenesis of HCCs, the MeCP2 shRNA and the control were transfected into HMCC‐97H and Huh7 cells. Using assays of wound healing, transwell invasion, tube formation, and spheroid sprouting, the inhibition of MeCP2 expression decreased the speed of HCC invasion, migration, and length of newly developing sprouts (Fig. 2E–H and Fig. S2E,F). Meanwhile, tail intravenous injection was used to confirm the function of MeCP2 in the metastasis of Huh7 cells *in vivo*. Compared with the LV‐negative control group, shMeCP2 suppressed tumor metastasis in the LV‐shMeCP2 group (Fig. 2I and Fig. S2G). In addition, western blotting was performed to explore MeCP2, HOXD3, HB‐EGF, EGFR, p‐MEK, and p‐ERK1/2 protein expression. From the gain‐of‐function of MeCP2, the expression levels of MeCP2, HOXD3, HB‐EGF, EGFR, p‐MEK, and p‐ERK1/2 were increased in MeCP2‐transfected HCCs. In contrast, the expression of MeCP2, HOXD3, HB‐EGF, EGFR, p‐MEK, and p‐ERK1/2 was inhibited in shMeCP2‐transfected HCCs (Fig. 2J), which strongly suggested that MeCP2 plays an essential role in tumor progression.

The article "MeCP2 drives hepatocellular carcinoma progression via enforcing HOXD3 promoter methylation and expression through the HB‐EGF/EGFR pathway" was retracted in 2024. Reasons: duplicated images; unreliable data; unreliable results or conclusions.

**Fig. 2:** MeCP2 expression activates HCC invasion, metastasis, and angiogenesis *in vitro* and *in vivo*. (A, B) Scratch wound and transwell invasion assays were applied to identify metastasis and invasion capability of HCCs after transfection of MeCP2‐Ctrl and MeCP2 in MHCC‐97H and Huh7 cells. Scale bar: 500 μm. (C) Effect of MeCP2 on tube formation of HUVECs. Scale bar: 50 μm. (D) The angiogenic ability of HUVECs after transfection with MeCP2 was examined by the 3D spheroid sprouting assay. Scale bar: 500 μm. (E–H) Scratch wound assay, transwell invasion assay, matrigel tube formation assay, and 3D spheroid sprouting assay of HCCs after suppressing MeCP2 expression. E, F, H, scale bar: 500 μm. G, scale bar: 50 μm. (I) Images of tumor metastasis from mice (*n* = 5). Inhibition of MeCP2 expression remarkably suppressed the migration of tumor to the mouse lung. Scale bar: 1 cm. (J) The expression of MeCP2, HOXD3, HB‐EGF, EGFR, p‐MEK, p‐ERK1/2, and GAPDH was detected by western blotting.

### 3.3 MeCP2 regulates HOXD3 by binding to the HOXD3 upstream promoter

Using the Pearson's and TCGA database assays, the expression of MeCP2 mRNA was significantly positively correlated with HOXD3 expression in HCC tissues (Fig. 3A). To further elucidate whether MeCP2 regulates the expression of HOXD3, the MeCP2 overexpression vector or MeCP2 shRNA was transfected into MHCC‐97H and Huh7 cell lines. The high expression of MeCP2 increased the expression of HOXD3, and silencing of MeCP2 resulted in the downregulated expression of HOXD3 (Fig. 3B). The JASPAR, VISTA, and UCSC genome browser tool databases were used to confirm the correlation between MeCP2 and HOXD3, and a presumed MeCP2‐binding site was found, which was located 0.3 kb upstream of the HOXD3 gene (Fig. 3C). ChIP‐PCR results revealed that MeCP2 directly binds to the promoter region of HOXD3 (Fig. 3D,E), and ChIP analysis of poly II A revealed binding to the GAPDH promoter as an internal reference (Fig. S3A). Moreover, a luciferase reporter assay was used to identify the role of MeCP2 in HOXD3 transcriptional activity in Huh7 cells. As shown in Fig. 3F, the overexpression of MeCP2 significantly increased the luciferase activity of HOXD3 WT in MeCP2‐transfected HCC cells compared with the control cells. It is worth noting that the promoter region of HOXD3 bound by MeCP2 is a CpG island, which contains four CpG sites.

**Fig. 3:** MeCP2 recruiting the CREB1 binds to the promoter of HOXD3 to active HOXD3 expression. (A) A correlation between MeCP2 and HOXD3 was identified by Pearson's *r*. (B) HOXD3 RNA expression in MHCC‐97H and Huh7 cells transfected with MeCP2‐Ctrl, MeCP2, shMeCP2‐Ctrl, and shMeCP2. (C) HOXD3‐binding sites in the promoter of HOXD3. (D) The interaction of MeCP2 with HOXD3 was revealed using ChIP assays. (E) qRT‐PCR was used with primers spanning the predicted MeCP2 of HOXD3. (F) Dual‐luciferase reporter assay was conducted to evaluate the luciferase activities of HOXD3 WT or HOXD3 Mut and MeCP2‐Ctrl or MeCP2 cotransfected in Huh7 cells. (G) HOXD3 expression was detected in HCCs treated with different doses of 5‐Aza. (H) Bisulfite sequencing was used to examine methylation levels of CpGs. (I) Schematic of MeCP2‐WT and various MeCP2 domain‐removed vectors. (J) Western blotting was performed to detect the expression of different MeCP2 types in HCCs. (K) A correlation between MeCP2 and the HOXD3 promoter was identified using ChIP analysis in HCCs transfected with different MeCP2 vectors. Simultaneous ChIP analysis of poly II A binding to GAPDH promoter as an internal reference. (L) The subcellular localization of exogenous proteins was detected by immunofluorescence staining in Huh7 cells. (M) The colocation of MeCP2 and CREB1 was tested by an immunofluorescence assay in HCCs. (N) The interaction with MeCP2 and HOXD3 was detected using Co‐IP (*n* = 3 per group. Significance was determined by Student's *t*‐test. Results are expressed as mean ± SEM.* *P* < 0.05, **P < 0.01.

The article "MeCP2 drives hepatocellular carcinoma progression via enforcing HOXD3 promoter methylation and expression through the HB‐EGF/EGFR pathway" was retracted in 2024. Reasons: duplicated images; unreliable data; unreliable results or conclusions.

DNA methylation in HOXD3 transcription was also investigated, and HCCs were treated with the methylation inhibitor 5‐azacytidine (5‐Aza) at different concentrations (Fig. 3G). The expression levels of HOXD3 were dependent on the inhibition of a methylation inhibitor, and the increasing dose of 5‐Aza induced lower expression of HOXD3. The BSP assay results revealed that there were two CpG sites bound by MeCP2, and their methylation levels were higher in Huh7 cells than in HL‐7702 cells (Fig. 3H). These experimental results suggest that methylation of the MeCP2‐binding site is important for controlling the transcription of HOXD3 in HCCs.

MeCP2 has two essential functional domains. One is the transcriptional repression domain (TRD), and the other is the methyl‐CpG binding domain (MBD). These two domains of MeCP2 have been studied in the regulation of gene function. All GFP‐tagged negative control vectors, MeCP2^WT^, and deletion mutants MeCP2^∆MBD^, MeCP2^∆TRD^, and MeCP2^∆TRD + NLS^ were constructed and transfected into HCCs, respectively. Western blotting (anti‐GFP), ChIP‐PCR (anti‐GFP), and immunofluorescence assays were performed to verify the exogenous gene expression and subcellular localization in HCCs (Fig. 3I–L and Fig. S3B,C). The MBD combined with the nuclear location sequence of MeCP2 was important for the occupation of HOXD3 in HCCs.

The article "MeCP2 drives hepatocellular carcinoma progression via enforcing HOXD3 promoter methylation and expression through the HB‐EGF/EGFR pathway" was retracted in 2024. Reasons: duplicated images; unreliable data; unreliable results or conclusions.

The cooperation between MeCP2 and CREB1 was investigated by immunofluorescence and Co‐IP assays (Fig. 3M,N), which confirmed the positive correlation between MeCP2 and HOXD3. MeCP2 recruited CREB1, contributing to an increase in invasion, migration, and angiogenesis *via* direct regulation of HOXD3 in HCCs.

### 3.4 HOXD3 induces angiogenesis of HCCs *in vitro*

In our previous study, HOXD3 functioned as an oncogene in HCC. HOXD3 induces metastasis and invasion of HCCs [18]. Considering that angiogenesis plays an essential role in tumor growth and migration, we further investigated the effect of HOXD3 on angiogenesis. Spheroid sprouting assays showed that HOXD3 markedly increased the length of newly developed sprouts. In contrast, inhibition of HOXD3 reduced the length of sprouts (Fig. 4A). In addition, tube formation assays showed that HOXD3 contributed to form tubular structures in HUVECs transfected with HOXD3 compared with control cells (Fig. 4B). Western blotting was performed to confirm the expression of HOXD3, HB‐EGF, EGFR, p‐MEK, and p‐ERK1/2 at the protein level. HOXD3, HB‐EGF, EGFR, p‐MEK, and p‐ERK1/2 expression levels were increased in HOXD3‐transfected HCCs. The low expression of HOXD3 contributed to the inhibition of HOXD3, HB‐EGF, EGFR, p‐MEK, and p‐ERK1/2 expression (Fig. 4C and Fig. S4A,B).

**Fig. 4:** Inhibition of HOXD3 rescues the effect of MeCP2 in HCCs. (A) 3D spheroid sprouting assay was used to identify the angiogenesis in HUVECs. Scale bar: 500 μm. (B) Tube formation assay was used to analyze the angiogenic ability in HUVECs transfected with HOXD3‐Ctrl, HOXD3, shHOXD3‐Ctrl, shHOXD3‐1, and shHOXD3‐2. Scale bar: 50 μm. (C) The expression of HOXD3, HB‐EGF, EGFR, p‐MEK, p‐ERK1/2, and GAPDH was detected by western blotting. (D–G) Wound healing assay, transwell assay, tube formation assay, and 3D spheroid sprouting assay were performed to measure the function of MeCP2 and HOXD3 on the angiogenic ability of cells after cotransfection with MeCP2 and shHOXD3‐1. D–F, scale bar: 500 μm. G, scale bar: 50 μm. (H) Western blotting analysis was used to examine HOXD3, HB‐EGF, EGFR, p‐MEK, p‐ERK1/2, and GAPDH expression in MHCC‐97H and Huh7 cells cotransfected with MeCP2 and shHOXD3‐Ctrl or shHOXD3‐1.

To understand whether MeCP2 regulates the migration, invasion, and angiogenesis of HCCs *via* HOXD3, shHOXD3 was cotransfected with MeCP2‐Ctrl or MeCP2 into MHCC‐97H and Huh7 cells. Inhibition of HOXD3 counterbalanced the tumor‐stimulating effect of␣MeCP2 in migration, invasion, and angiogenesis of HCCs, indicating that increasing MeCP2 expression promotes metastasis, invasion, and angiogenesis of HCCs. In contrast, the inhibition of HOXD3 suppressed the effects of MeCP2 on MHCC‐97H and Huh7 cells (Fig. 4D–H and Fig. S4C–F). These results further suggest that MeCP2 is a tumor activator that directly targets HOXD3.

The article "MeCP2 drives hepatocellular carcinoma progression via enforcing HOXD3 promoter methylation and expression through the HB‐EGF/EGFR pathway" was retracted in 2024. Reasons: duplicated images; unreliable data; unreliable results or conclusions.

### 3.5 HOXD3 binds to the promoter of HB‐EGF to activate the metastasis of HCCs

The results of TCGA and GTEX analysis assays showed that HB‐EGF was significantly upregulated in HCC cancer samples (*P* < 0.001; Fig. 5A). The RNA‐Seq assay was used to study the molecular mechanisms induced by HOXD3, which regulates the function of HB‐EGF in HCC invasion, migration, and angiogenesis. A total of 112 upregulated genes and 56 downregulated genes were confirmed. Among the upregulated genes, HB‐EGF was identified (Fig. 5B). All gene enrichment assays showed that the upregulation of HOXD3 in Huh7 cells was associated with the modification of cell angiogenesis and migration (Fig. 5C). In addition, the TCGA database revealed that HB‐EGF expression was positively correlated with MeCP2 expression (*P* < 0.001, *r* = 0.40; Fig. 5D). HB‐EGF was negatively associated with the survival rate of the clinical samples (Fig. 5E and Fig. S5A–C), and the expression of HB‐EGF induced a lower DSS (*P* = 0.036), PFI (*P* = 0.046), and OS (*P* = 0.013) of HCC. HB‐EGF expression in liver cancer tissues was identified by qRT‐PCR, western blotting, and IHC. Compared with normal tissues, HB‐EGF expression was promoted at the RNA and protein levels (Fig. 6A–C). In addition, the upregulation of HB‐EGF was associated with the histology of HCC samples (Table 1). Using assays of wound healing, transwell invasion, and tube formation, the overexpression of HB‐EGF increased the speed of HCC invasion and migration (Fig. 6D–F). In line with the bioinformatics results, the expression of HB‐EGF was positively correlated with MeCP2 and HOXD3 (Fig. 6G), and the expression of MeCP2 or HOXD3 induced the expression of HB‐EGF in HCCs (Fig. 6H). The UCSC genome browser tool, PROMO, JASPAR database, and ChIP‐PCR experiments were used to further confirm the relationship between HOXD3 and HB‐EGF. The results showed that two presumed HOXD3‐binding sites were located 3.8 and 4.5 kb upstream of the HB‐EGF gene, respectively (Fig. 6I,J). Double‐luciferase reporter assays were performed to examine the role of HOXD3 in HB‐EGF transcriptional regulation. In contrast to HOXD3‐control‐transfected HCCs, HB‐EGF activity was remarkably increased in HOXD3‐transfected cells (Fig. 6K), suggesting that HOXD3 induced migration, invasion, and angiogenesis of HCCs by directly regulating HB‐EGF transcription in MHCC‐97H and Huh7 cells (Fig. 7).

The article "MeCP2 drives hepatocellular carcinoma progression via enforcing HOXD3 promoter methylation and expression through the HB‐EGF/EGFR pathway" was retracted in 2024. Reasons: duplicated images; unreliable data; unreliable results or conclusions.

**Fig. 5:** The relationship between HOXD3 and HB‐EGF was examined by bioinformatics data. (A) HB‐EGF expression in normal (*n* = 160) and HCC tissues (*n* = 371) data from TCGA (B) RNA‐Seq results showed that HOXD3 induced the expression of HB‐EGF. (C) GO data indicated that HB‐EGF participated in cell migration and angiogenesis. (D) TCGA and GTEX showed the relationship between MeCP2 and HB‐EGF by the Pearson correlation coefficient. (E) The higher expression of HB‐EGF was correlated with a lower survival rate (*n* = 3 per group. Significance was determined by Student's *t*‐test. All data are mean ± SD. **P < 0.01).

**Fig. 6:** HOXD3 binds to the promoter region of HB‐EGF and induces the expression of HB‐EGF. (A) HB‐EGF expression in 36 pairs of liver cancer tissues and normal tissues at the RNA level. Data are shown as mean ± SD. (B, C) HB‐EGF expression at the protein level in liver cancer tissues versus normal tissues was examined by performing IHC and western blotting assays. (D–F) Wound healing, transwell invasion, and tube formation assays were used to examine HCC metastasis and invasion capability after transfection of HB‐EGF‐Ctrl and HB‐EGF in MHCC‐97H and Huh7 cells. (G) Pearson's r was performed to identify the interaction between HOXD3 and HB‐EGF, MeCP2, and HB‐EGF. (H) HB‐EGF expression in MHCC‐97H and Huh7 cells was confirmed by qRT‐PCR following overexpression MeCP2/HOXD3 expression and inhibition of MeCP2/HOXD3. Data are shown as mean ± SEM. (I) Schematic of the two presumed HOXD3 response sites on the HB‐EGF promoter (top). The relationship between HOXD3 and HB‐EGF was revealed by using ChIP assays (down). (J) RT‐PCR was used with primers spanning the predicted HOXD3 of HB‐EGF. The error bar was SEM. (K) Luciferase activity relative to the Renilla control was examined in Huh7 cells. The error bar was SEM. (*n* = 3 per group. Significance was determined by Student's *t*‐test. *P < 0.05, **P < 0.01).

**Fig. 7:** Proposed model of MeCP2 binding to the HOXD3 upstream methylated promoter *via* the HB‐EGF–EGFR‐ERK1/2 signaling pathway to regulate the invasion, metastasis, and angiogenesis of HCC.

## 4 Discussion

Initially, the critical roles of homeobox genes are found in tissue differentiation during embryonic development, cell differentiation, and essential processes of eukaryotic cell life [21, 22]. In mammals, 39 HOX genes have been divided into four paralogous clusters. HOXA, HOXB, HOXC, and HOXD are located on various chromosomes [23]. Recently, a large number of aberrant HOX genes have been identified in cancer [24, 25]. In ovarian cancer, upregulated HOXA13, B6, C13, D1, and D13 are associated with poor clinical outcomes [26]. The HOXB cluster is performed to overcome the limitations of tamoxifen‐resistant cancer treatments in breast cancer and is a potential therapeutic target [27]. In the HCC research field, our previous studies revealed that HOXD3 in HCC cell lines and liver cancer samples showed higher expression than normal liver cells and tissues, which is an oncogene in tumorigenesis [18]. Combined with our previous research and the current study, the overexpression of HOXD3 promoted the invasion, migration, tube formation, and sprouting angiogenesis of HCC cells (Fig. 4). Using bioinformatics and weighting and scoring analysis assays, the hypermethylated differentially methylated region was detected in the promoter region of HOXD3 in HCC; however, HOXD3 expression in HCC samples was higher than that in normal tissues [28]. Consistent with the above results, the expression of HOXD3 was dependent on the inhibition of a methylation inhibitor, and the increasing dose of 5‐Aza induced lower expression of HOXD3 (Fig. 3). Interestingly, the results differed from the conventional theory that the hypermethylated promoter region of the gene caused the lower expression. To further elucidate the underlying mechanism, we used bioinformatics assays and bisulfite sequencing PCR to test the methylation level in the promoter of HOXD3 in HCC cells and normal liver cells. Four methylated CpG sites were found in the promoter of HOXD3, which was located 0.3 kb upstream of HOXD3. The methylation level of the two CpG sites in Huh7 cells was higher than that in normal liver HL‐7702 cells. Meanwhile, the two hypermethylated CpG sites were located in the HOXD3 promoter region, which was bound by MeCP2 (Fig. 3).

The article "MeCP2 drives hepatocellular carcinoma progression via enforcing HOXD3 promoter methylation and expression through the HB‐EGF/EGFR pathway" was retracted in 2024. Reasons: duplicated images; unreliable data; unreliable results or conclusions.

MeCP2 is a classic methylated‐DNA‐binding protein, which was initially recognized as an epigenetic regulator that participates in the regulation of functions in the brain and neurons [29, 30]. MeCP2 contains two crucial domains, TRD and MBD. MBD binds to methylated cytosine in the DNA sequence of CpGs. In the present study, different vectors (MeCP2, MeCP2^∆MBD^, MeCP2^∆TRD^, and MeCP2^∆TRD + NLS^) were transfected into the HCCs to confirm which domain was responsible for MeCP2 binding to the promoter region of HOXD3. Figure 3 indicates that MBD and the NLS of MeCP2 are important for HOXD3 occupation. Meanwhile, MeCP2 may play a role as a transcriptional activator and bind to methylated CpGs, and thereby recruit CREB1 to regulate gene expression [31]; this is corroborated by our results of CO‐IP and immunofluorescence assays, and MeCP2 combined with CREB1 targeted the promoter hypermethylation region of HOXD3 to facilitate invasion, migration, and angiogenesis of HCCs (Fig. 3). Using the TCGA database and GTEX assays, the expression of CREB1 in HCC samples was higher than that in normal tissues (*P* < 0.001). In addition, the expression of CREB1 was associated with the pathologic stage and T of HCC patient specimens (*P* = 0.043 and 0.046, respectively).Furthermore, the expression of CREB1 was related to OS (*P* = 0.021), PFI (*P* = 0.011), DFI (*P* = 0.017), and DSS (*P* = 0.0064) in HCC patients, which was positively correlated with MeCP2 expression (*P* < 0.001, *r* = 0.47) (Fig.␣S6). As far as we know, it is the first time that the correlated MeCP2, CREB1 with HOXD3 is demonstrated in the promotion of HCC invasion, migration, and angiogenesis.

To date, the function of MeCP2 in tumor progression has not been extensively investigated, and an increasing amount of evidence supports that MeCP2 is a tumor activator in cancer development. MeCP2 facilitates breast cancer progression by activating ubiquitination‐mediated P53 degradation by suppressing RPL5/RPL11 transcription [32]. Luo and Ge [33] showed that MeCP2 promotes colorectal cancer metastasis by modulating ZEB1 transcription. In pancreatic cancer, MeCP2 drove the Furin/TGF‐β1/Smad axis to increase epithelial–mesenchymal transition in pancreatic cancer cells [34]. In our present study, TCGA and GTEX data revealed that MeCP2 expression was remarkably higher in HCC tissues and was correlated with patients' survival rate; these results were confirmed in our 36 paired HCC tissues. Meanwhile, the expression of MeCP2 was related to the clinical pathologic stage and T (Fig. 1). Using transwell invasion, tube formation, scratch wound, and spheroid sprouting assays, we found that MeCP2 induced the invasion, migration, and angiogenesis of HCCs by targeting the promoter of HOXD3. Furthermore, the inhibition of HOXD3 expression reversed the tumor biological function‐increasing effect of MeCP2 on HCCs (Fig. 2), suggesting that MeCP2 is a key oncogene in HCC progression.

Bioinformatics, RNA‐Seq, RT‐PCR, ChIP‐PCR, luciferase reporter, and western blotting assays were performed to identify the role of HOXD3 in the regulatory mechanism of HCCs, and Fig. 6 shows that HOXD3 binds to the promoter region of HB‐EGF. Previous studies have shown that HB‐EGF is involved in tumor progression [35, 36, 37]. HB‐EGF can bind to the receptors HER1 (EGFR/ErbB1) and HER4 (ErbB4) by activating the downstream cell signaling pathways RAS‐RAF‐MEK‐ERK, JAK‐STAT, PLCγ‐PKC‐CAMK, and PIL3‐AKT‐mTOR to regulate cell proliferation, angiogenesis, and migration, thus facilitating metastasis of the tumors [38]. Combined with the TCGA and GTEX databases, the upregulation of HB‐EGF in liver cancer tissues was associated with the survival of HCC patients, which is consistent with previous research [8]. High expression of HB‐EGF increased the invasion and migration of HCC cells. We have also revealed that HOXD3 directly targets the promoter of HB‐EGF and induces the activation of HB‐EGF (Fig. 5).

The article "MeCP2 drives hepatocellular carcinoma progression via enforcing HOXD3 promoter methylation and expression through the HB‐EGF/EGFR pathway" was retracted in 2024. Reasons: duplicated images; unreliable data; unreliable results or conclusions.

## 5 Conclusions

In summary, the expression of MeCP2, HOXD3, and HB‐EGF was increased in HCC, and the activation of genes was correlated with poor survival rates. This study is the first to demonstrate that MeCP2 recruiting CREB1 enforces HOXD3 expression by directly targeting the promoter hypermethylation sites of HOXD3 *via* the HB‐EGF cell signaling pathway to induce the invasion, migration, and angiogenesis of HCC *in vitro* and *in vivo*. Our findings suggest that MeCP2/HOXD3/HB‐EGF acts as an attractive candidate for targeted therapeutics and may serve as a potentially novel biomarker.

## Conflict of interest

The authors declare no conflict of interest.

## Author contributions

LW contributed to study concept and design. YY, DT, YQ, CG, and BG contributed to acquisition of data. YG, JY, LL, LZ, and JZ contributed to analysis and interpretation of data. LW drafted the manuscript. CH contributed to critical revision of the manuscript for important intellectual content. XW contributed to administrative, technical, and material support. All authors read and approved the final manuscript.

## Ethical standards

The study was approved by the Institutional Research Ethics Committee of Xi'an Jiaotong University. Informed consent was obtained from each patient before collecting samples.

### Peer Review

The peer review history for this article is available at https://publons.com/publon/10.1002/1878‐0261.13019.

## Supporting information


**Fig.␣S1**. The expression of MeCP2 induces the lower survival rate.

**Fig.␣S2**. The function of MeCP2 on HCCs invasion, migration and angiogenesis.

**Fig.␣S3**. The expression and location of different MeCP2 domain deletion vectors in HCCs.

**Fig.␣S4**. MeCP2 regulates biological function of HCCs *via* directly targeting HOXD3.

**Fig.␣S5**. The expression of HB‐EGF induces the lower survival rate.

**Fig.␣S6**. The function of CREB1 on HCCs progression.

**Table␣S1**. Primers and oligonucleotides used in this work.

## Data Availability

All experimental data during this research are included in the published article and its supplementary files. The datasets and materials in this study are available on reasonable request from corresponding authors.
